The article "Genetic Analysis of Invasive Aedes albopictus Populations in Los Angeles County, California and Its Potential Public Health Impact" was published in 2013. Journal: PLoS One.

# Genetic Analysis of Invasive *Aedes albopictus* Populations in Los Angeles County, California and Its Potential Public Health Impact

**DOI:** 10.1371/journal.pone.0068586

**Published:** 2013-07-05

**Authors:** Daibin Zhong, Eugenia Lo, Renjie Hu, Marco E. Metzger, Robert Cummings, Mariangela Bonizzoni, Kenn K. Fujioka, Teresa E. Sorvillo, Susanne Kluh, Sean P. Healy, Chris Fredregill, Vicki L. Kramer, Xiaoguang Chen, Guiyun Yan

**Affiliations:** 1 Program in Public Health, College of Health Sciences, University of California Irvine, Irvine, California, United States of America; 2 Vector-Borne Disease Section, California Department of Public Health, Ontario, California, United States of America; 3 Orange County Vector Control District, Orange, California, United States of America; 4 San Gabriel Valley Mosquito and Vector Control District, West Covina, California, United States of America; 5 Greater Los Angeles County Vector Control District, Santa Fe Springs, California, United States of America; 6 Monmouth County Mosquito Extermination Commission, Tinton Falls, New Jersey, United States of America; 7 Harris County Public Health and Environmental Services, Mosquito Control Division, Houston, Texas, United States of America; 8 Department of Parasitology, School of Public Health and Tropical Medicine, Southern Medical University, Guangzhou, People’s Republic of China; Centro de Pesquisas René Rachou, Brazil

## Abstract

The Asian tiger mosquito, *Aedes albopictus*, is an anthropophilic aggressive daytime-biting nuisance and an efficient vector of certain arboviruses and filarial nematodes. Over the last 30 years, this species has spread rapidly through human travel and commerce from its native tropical forests of Asia to every continent except Antarctica. In 2011, a population of Asian tiger mosquito (*Aedes albopictus*) was discovered in Los Angeles (LA) County, California. To determine the probable origin of this invasive species, the genetic structure of the population was compared against 11 populations from the United States and abroad, as well as preserved specimens from a 2001 introduction into California using the mitochondrial cytochrome c oxidase 1 (CO1) gene. A total of 66 haplotypes were detected among samples and were divided into three main groups. *Aedes albopictus* collected in 2001 and 2011 from LA County were genetically related and similar to those from Asia but distinct from those collected in the eastern and southeastern United States. In view of the high genetic similarities between the 2001 and 2011 LA samples, it is possible that the 2011 population represents in part the descendants of the 2001 introduction. There remains an imperative need for improved surveillance and control strategies for this species.

The article "Genetic Analysis of Invasive Aedes albopictus Populations in Los Angeles County, California and Its Potential Public Health Impact" was published in 2013. Journal: PLoS One.

## Introduction

The Asian tiger mosquito *Aedes albopictus* (Skuse) is currently the most invasive mosquito species in the world. Over the last 30 years, this species has spread rapidly through human travel and commerce from its native tropical forests of Asia to every continent except Antarctica [1], [2]. Adult females are anthropophilic aggressive daytime-biting nuisances and efficient vectors of certain arboviruses and filarial nematodes including dengue, chikungunya, and dog heartworm [3], [4]. Although *Ae. albopictus* is a less competent vector of arboviruses than its congeneric species *Ae. aegypti* (L.) [1], its importance in the transmission of endemic dengue in rural Asia is well elucidated [5]. Recent outbreaks of chikungunya and dengue in Hawai’i, Mauritius, Gabon, Madagascar, and La Reunion [6] and the first endogenous transmission of chikungunya and dengue in Europe [7], [8] sustained by *Ae. albopictus* further demonstrate the increasing public health impact of this species worldwide.

The first clearly established population of *Ae. albopictus* in the continental United States (U.S.) was discovered in Harris County, Texas, during the summer of 1985 [9]. The most likely route of its introduction and spread was through the unintentional transport of dormant eggs in automobile tires imported from Asia [3], [10]. In less than two decades, the known geographic range of *Ae. albopictus* expanded to much of the eastern U.S., including at least 911 counties in 25 states [11]. In California, cargo shipments from the South Pacific region introduced *Ae. albopictus* at least four times between 1946 and 2004 [12]. The most severe and widespread infestations in the state were discovered in 2001 when *Ae. albopictus* was imported from mainland China in trans-oceanic shipments of “lucky bamboo” (*Dracaena* spp.) packaged in standing water. Distribution of these plants to wholesale nurseries throughout California resulted in 15 localized infestations in six counties [13]. Follow-up surveys in 2002 revealed that *Ae. albopictus* had survived the winter at some of those sites, but no evidence was subsequently found to suggest that populations had become established [13], [14]. The combination of low rainfall, low humidity, and high temperatures during summer in California may have posed a major obstacle to successful colonization by this species [2], [15], [16].

In early September 2011, *Ae. albopictus* was discovered in the City of El Monte, Los Angeles County, following a request from a citizen for vector control service [17]. Enhanced surveillance by local vector control agencies found this mosquito throughout most of the city and in a portion of the neighboring City of South El Monte. Despite a concerted campaign to eradicate *Ae. albopictus*, the population survived and reemerged throughout the infested area in May of 2012. The source of this inland population of *Ae. albopictus* was uncertain since a connection to international commerce was lacking. Possible sources of the infestation included an introduction from other regions of the U.S. mainland where *Ae. albopictus* is established, importation from Hawai’i or abroad, or surviving mosquitoes from past introductions. Elucidating the origin of these mosquitoes could identify new invasion pathways and the potential for continued expansion. We compared samples of this newly-discovered population of *Ae. albopictus* to preserved specimens from past introductions and populations from other regions of the U.S. and other countries. We also assessed the potential impact to public health in California of an established population of *Ae. albopictus*.

The article "Genetic Analysis of Invasive Aedes albopictus Populations in Los Angeles County, California and Its Potential Public Health Impact" was published in 2013. Journal: PLoS One.

## Materials and Methods

### Ethics Statement

No permits were required for this study. Residents consented at all properties where mosquitoes were collected. No sites were protected by law and this study did not involve endangered or protected species.

### Mosquito Samples

*Aedes albopictus* were collected as larvae or adults from 11 localities in the U.S. and around the world in 2011 (Table 1). Samples were collected from the native home range (China, Japan, Taiwan, and Singapore), from non-native areas with established populations (Hawai’i, New Jersey, Texas, and Italy), and from the City of El Monte, Los Angeles County, California. In addition, preserved specimens that were collected in the City of Rowland Heights, Los Angeles County, in 2001 were included in the study. A total of 346 mosquitoes were tested with each locality represented by 15–36 individual specimens. All specimens were confirmed as *Ae. albopictus* using PCR with species-specific primers for the ribosomal internal transcribed spacer (ITS1 and ITS2) and 18S rDNA regions [18].

**Table 1:** Location of specimen collection sites of *Aedes albopictus* mosquitoes analyzed.

Site ID	Name	Origin	Geographic coordinate(latitude, longitude)	Year ofcollection	Life-stagesanalyzed	Specimensgenotyped
**1**	GZ	Guangzhou city, Guangdong, China	23.128521,113.246899	2011	larvae	32
**2**	XM	Xiamen city, Fujian, China	24.480275,118.13736	2011	adult	29
**3**	JS	Wuxi city, Jiangsu, China	31.566145,120.303027	Lab strain*	adult	30
**4**	TW	Xinzhu, Hsinchu, Taiwan	24.803946,120.964687	2011	adult	30
**5**	JP	Nagasaki city, Japan	32.750286,129.877667	2011	adult	15
**6**	SG	Helios Block, Serangoon, Singapore	1.362176,103.870239	2011	adult	36
**7**	IT	Arco, Trentino, Italy	45.917826,10.886866	2011	adult	32
**8**	LA01	Los Angeles County, California, United States	33.976124,−117.905339	2001	adult	15
**9**	LA11	Los Angeles County, California, United States	34.059792, −118.040167	2011	adult & larvae	34
**10**	NJ	Monmouth County, New Jersey, United States	40.433163, −74.199588	2011	adult	30
**11**	TX	Harris County, Texas, United States	29.775183, −95.31025	2011	adult	31
**12**	HW	O’ahu, Hawai’i, United States	21.447317, −158.014812	2011	adult	32

* Laboratory-maintained strain cultured from local field collection in Wuxi, China.

The article "Genetic Analysis of Invasive Aedes albopictus Populations in Los Angeles County, California and Its Potential Public Health Impact" was published in 2013. Journal: PLoS One.

### Mitochondrial DNA Analysis

Total DNA was extracted from a single mosquito leg of each specimen using the Fast Tissue-to-PCR Kit (Fermentas Inc., Glen Burnie, MA) following the methods of Zhong et al. [19]. The mitochondrial gene cytochrome c oxidase subunit 1 (CO1) was used to examine sequence polymorphism among mosquito samples. DNA samples were amplified with the following two sets of primers: 1454F (5′ GGTCAACAAATCATAAAGATATTGG 3′) and 2160R (5′ TAAACTTCTGGATGACCAAAAAATCA 3′); 2027F (5′ CCCGTATTAGCCGGAGCTAT 3′) and 2886R (5′ ATGGGGAAAGAAGGAGTTCG 3′). A total of 23 µl reaction mix containing 3 µl of template DNA, 0.5 mM MgCl_2_, 0.2 mM dNTP, 10 pmol of each primer and 0.5 U of Taq polymerase (Qiagen) was used in each PCR, and amplification was performed in a Bio-Rad MyCycler Thermal Cycler. PCR cycles involved an initial denaturing step at 94°C for 3 min, then 35 cycles of 94°C for 30 s, 55°C for 30 s, and 72°C for 1 min. An additional extension was performed at 72°C for 6 min. Products of PCR were visualized on 1% agarose gels and then purified and sequenced directly using primers 2160R and 2027F with ABI Big Dye Terminator Cycle Sequencing Kit.

### Data Analysis

The CO1 gene sequences from 346 mosquitoes were aligned using BioEdit, and then edited manually with Sequence Alignment Editor version 1.d1 (SE-Al) [20]. The number of polymorphic sites, haplotype diversity (*Hd*), and nucleotide diversity (π) within each of the sites were determined using DnaSP version 4.10.1 [21]. To determine the relationships among the samples, haplotypes based on sequence variation were identified and then used to construct a network among the defined haplotypes using a statistical parsimony algorithm implemented in TCS version 1.13 [22]. Haplotypes were connected when the parsimony had a probability of at least 0.95 of being true as established by coalescence theory, starting with the shortest distance until all haplotypes were joined or the distance exceeded the parsimony limit [22].

To examine genetic structuring of individuals, a model-based Bayesian analysis was performed on the basis of nucleotide variation using STRUCTURE version 2.2 under varying assumptions on Hardy–Weinberg (HW) and linkage equilibriums [23]. The number of clusters (*K*) was determined by simulating a range of *K* values from 1 (no genetic differentiation among all sites) to 12 (all sites are genetically differentiated from one another). The posterior probability of each value was then used to detect the modal value of Δ*K*, a quantity related to the second order rate of change with respect to *K* of the likelihood function [24]. Posterior probability values were estimated using a Markov Chain Monte Carlo (MCMC) method and 1,000,000 iterations of each chain following the 100,000 iteration burn-in period were performed, as recommended by Pritchard *et al*. [23]. Each MCMC chain for each value of *K* was run five times with the ‘independent allele frequency’ option that allows individuals with ancestries in more than one group to be assigned into one cluster. Individuals were partitioned into multiple groups according to the membership coefficient (Q) that ranges from 0 (lowest affinity to a group) to 1 (highest affinity to a group) across the *K* groups. The partitioning of clusters was visualized using the program DISTRUCT [25].

The article "Genetic Analysis of Invasive Aedes albopictus Populations in Los Angeles County, California and Its Potential Public Health Impact" was published in 2013. Journal: PLoS One.

Genetic distance matrices were calculated using Kimura two-parameter distance [26] with Arlequin version 3.5 [27]. Analysis of molecular variance (AMOVA) [28] was conducted to determine the distribution of genetic variation within and among populations, and significance level was tested with the Markov chain method (n = 100,000). Genetic differentiation estimates were calculated using population pairwise *F*_ST_ [29] statistics. Null hypothesis of genetic homogeneity was assessed by 10,000 replications and sequential Bonferroni corrections [30] for multiple comparisons were applied to all comparisons. Deviations from selective neutrality were tested by Fu’s *Fs* statistics [31] and Tajima’s *D* [32]. Neutrality test was used to examine recent population expansion when the null hypothesis of neutrality was rejected due to significant negative values. For the two populations from LA (LA01 and LA11), mismatch analysis was conducted using Arlequin and DnaSP under the model of population expansion. The overall validity of the estimated demographic model was evaluated by the tests of Harpending's raggedness index (*Hri*) [33] and the sum of squared differences (SSD) [34].

## Results

### Sequence Variation and Haplotype Network

The mitochondrial CO1 gene gave a total aligned length of 1,433 bp in which 35 variable sites were observed and 33 of them were parsimony informative (Table 2, Table S1). Haplotype diversity (*H_d_*) ranged from 0.37 in the laboratory strain from Jiangsu, China to 0.83 in preserved specimens from Los Angeles County, California, collected in 2001 (LA01). Nucleotide diversity (π) ranged from 0.06 in specimens from Guangzhou and Taiwan to 0.30 in specimens collected in Singapore. Overall, samples from southern China (XM) and southern California (LA01) showed the highest diversity, whereas the laboratory strain (JS) showed the lowest diversity, followed by specimens from the City of El Monte in Los Angeles County, California, collected in 2011 (LA11) and from Monmouth County, New Jersey (NJ).

The article "Genetic Analysis of Invasive Aedes albopictus Populations in Los Angeles County, California and Its Potential Public Health Impact" was published in 2013. Journal: PLoS One.

**Table 2:** Haplotype and nucleotide diversity of the mitochondrial cytochrome c oxidase 1 (CO1) gene.

Site ID	Sample size	# of variable sites	# of parsimony informative sites	# of haplotypes	Haplotype diversity (± SD)	Nucleotide diversity (×10^2^)	Tajima’s *D*	Fu’s *Fs*
**GZ**	32	6	3	6	0.59±0.09	0.06	−1.06	**−**2.45*
**XM**	29	11	6	11	0.82±0.05	0.17	−0.66	**−**3.82*
**JS**	30	3	3	2	0.37±0.08	0.08	1.10	3.70
**TW**	30	8	2	8	0.59±0.10	0.06	−1.80*	**−**4.85**
**JP**	15	3	2	3	0.59±0.07	0.09	0.77	1.26
**SG**	36	11	11	11	0.74±0.06	0.30	1.45	**−**0.71
**IT**	32	7	7	11	0.81±0.06	0.15	0.33	**−**4.21*
**LA01**	15	9	8	6	0.83±0.06	0.23	0.22	0.20
**LA11**	34	8	5	6	0.51±0.09	0.14	−0.26	0.24
**NJ**	30	4	4	5	0.54±0.10	0.07	**−**0.14	**−**0.75
**TX**	31	12	11	9	0.72±0.08	0.15	**−**1.14	**−**2.21
**HW**	32	8	6	8	0.69±0.07	0.11	**−**0.92	**−**2.51

Corresponding Tajima’s *D* and Fu’s *Fs* values are also indicated. GZ: Guangzhou; XM: Xiamen; JS: Jiangsu; TW: Taiwan; JP: Japan; SG: Singapore; IT: Italy; LA01: Los Angeles 2001; LA11: Los Angeles 2011; NJ: New Jersey; TX: Texas; and HW: Hawai’i.

* P<0.05;

** P<0.01.

Sixty-six haplotypes were detected (Table 2, Table S1, GenBank accession nos. KC690896-KC690961) and distinguished from each other by four to eight mutation steps in the phylogenetic network (Fig. 1). Samples collected in Italy (IT) and Southeast Asia (SG and XM) contained the highest number of haplotypes (Table 2). Most of these haplotypes were unique and generally connected with each other, except those of Singapore that were found separated as two distant groups (Fig. 1). CO1 haplotypes can be divided into three main groups: Group 1 contains mainly haplotypes from Singapore (SG; yellow) and Los Angeles County, California (LA01; orange); Group 2 contains haplotypes from Guangzhou, China (GZ; red), Taiwan (TW; purple), Japan (JP; pink), and Hawai’i (HW; black); and Group 3 contains mainly haplotypes from Xiamen, China (XM; green) and Los Angeles County, California (LA01 and LA11; orange). Haplotypes of group 3 were further connected to haplotypes from Europe and the eastern and central U.S. (Fig. 1). Specimens from two sites in the continental U.S., Monmouth County in New Jersey and Harris County in Texas, shared two haplotypes with the Italian samples. Haplotypes of these three sites were all connected to one another, indicative of their close genetic relatedness. In contrast, haplotypes from Los Angeles County (LA01 and LA11) were distinctively different from the New Jersey and Texas samples, but closely related to haplotypes of Singapore and southern China (GZ, XM and JS; Fig. 1).

The article "Genetic Analysis of Invasive Aedes albopictus Populations in Los Angeles County, California and Its Potential Public Health Impact" was published in 2013. Journal: PLoS One.

**Figure 1:** Phylogenetic network of 66 mitochondrial haplotypes of CO1 gene in *Aedes albopictus* from 11 localities. Localities are indicated by different color (bottom-right) and samples of LA01 and LA11 are labeled by crosses and asterisks, respectively. Sizes of circles are approximately proportional to the number of individuals with the given haplotype. GZ: Guangzhou; XM: Xiamen; JS: Jiangsu; TW: Taiwan; JP: Japan; SG: Singapore; IT: Italy; LA01: Los Angeles 2001; LA11: Los Angeles 2011; NJ: New Jersey; TX: Texas; and HW: Hawai’i.

### Genetic Clustering of Samples

The optimal partitioning of all samples is obtained for *K* = 6 with structure analysis. The pie charts in Fig. 2 show the proportional membership coefficient of individuals in the twelve *Ae. albopictus* populations studied. The largest membership coefficient value (Q), or the proportion of individuals assigned to a cluster, were high for New Jersey and Texas samples (Q >0.74), suggesting a strong affinity to be included in a single cluster (cluster 4). This cluster was shared with some of the individuals from Italy, consistent with the results obtained in the network analysis (Fig. 1). Individuals from southern China (GZ, XM and JS) and Taiwan constituted three major genetic clusters (clusters 2, 3, and 6; Fig. 2). These clusters were also shared with individuals from Los Angeles County (LA01 and LA11) as well as from Hawai’i, suggesting a temperate Asian origin of these samples.

**Figure 2:** Bayesian cluster analysis using STUCTURE program. **A)** Pie charts showing the composition of proportional membership coefficient of *Aedes albopictus* individuals within the 6 clusters identified by the Bayesian analyses; and **B)** color code of respective clusters and membership coefficient values for the *Aedes albopictus* populations studied. The coefficient values above 0.20 are highlighted in bold. GZ: Guangzhou; XM: Xiamen; JS: Jiangsu; TW: Taiwan; JP: Japan; SG: Singapore; IT: Italy; LA01: Los Angeles 2001; LA11: Los Angeles 2011; NJ: New Jersey; TX: Texas; and HW: Hawai’i.

### Population Genetic Structure

AMOVA found a significant overall population structure in *Ae. albopictus* (*F*_ST_ = 0.35, *p*<0.001). The majority of genetic variation (65%) was within-populations, whereas approximately 35% was among-population. Pairwise *F*_ST_ values ranged from 0.09 (JS and IT) to 0.69 (GZ and NJ) (Table 3). No genetic differentiation was observed between the Los Angeles County samples collected in 2001 and 2011 (*F*_ST_ = 0.11, *p*>0.05). Samples collected in 2001 and 2011 from Los Angeles County exhibited a large genetic differentiation from samples from New Jersey and Texas (*p*<0.001), suggesting they are not likely the origin of the Los Angeles County samples. Tajima’s *D* values for LA01 and LA11 are 0.22 and **−**0.26, respectively, and these values are not statistically significant (*p*>0.05). Tajima’s *D* value for all other studied localities, with the exception of TW (*D* = **−**1.80, *p*<0.05), are also not statistically significant (Table 2), indicating that most of the populations are in genetic equilibrium and consistent with the neutral mutation hypothesis [32]. Likewise, Fu’s *Fs* test for the two Los Angeles populations was not significant and rejected the population expansion/bottleneck model (Table 2). The bimodal mismatch distribution and significance of SSD (P<0.05) values indicated a poor fit for the stepwise growth model, suggesting a relative constant population size, although the test of *Hri* for LA11 was not significant (P>0.05) (Fig. 3).

The article "Genetic Analysis of Invasive Aedes albopictus Populations in Los Angeles County, California and Its Potential Public Health Impact" was published in 2013. Journal: PLoS One.

**Figure 3:** Observed and expected mismatch distributions showing the frequencies of pairwise differences. The observed distributions (blue bars) are compared for their goodness-of-fit to a Poisson distribution under a model of sudden expansion illustrated by the overlaid curve (red dots and solid lines).

**Table 3:** Pairwise genetic differentiation (*F*_ST_) between *Ae. albopictus* populations.

Pop	GZ	XM	JS	TW	JP	SG	IT	LA01	LA11	NJ	TX	HW
**GZ**	–											
**XM**	0.40*	–										
**JS**	0.14	0.34*	–									
**TW**	0.46*	0.31*	0.33*	–								
**JP**	0.27	0.41*	0.28	0.53*	–							
**SG**	0.34*	0.35*	0.30*	0.33*	0.17	–						
**IT**	0.18*	0.30*	0.09	0.23*	0.25*	0.27*	–					
**LA01**	0.26*	0.16	0.23	0.19*	0.29*	0.19	0.17	–				
**LA11**	0.13	0.23*	0.12	0.23*	0.24	0.26*	0.12	0.11	–			
**NJ**	0.69*	0.52*	0.59*	0.53*	0.69*	0.46*	0.34*	0.47*	0.53*	–		
**TX**	0.53*	0.40*	0.46*	0.37*	0.53*	0.38*	0.26*	0.29*	0.38*	0.12*	–	
**HW**	0.26*	0.41*	0.26*	0.43*	0.33*	0.36*	0.25*	0.30*	0.23*	0.63*	0.51*	–

GZ: Guangzhou; XM: Xiamen; JS: Jiangsu; TW: Taiwan; JP: Japan; SG: Singapore; IT: Italy; LA01: Los Angeles 2001; LA11: Los Angeles 2011; NJ: New Jersey; TX: Texas; and HW: Hawai’i.

* Asterisks indicate significant values after Bonferroni correction (P<0.05).

The article "Genetic Analysis of Invasive Aedes albopictus Populations in Los Angeles County, California and Its Potential Public Health Impact" was published in 2013. Journal: PLoS One.

## Discussion

*Aedes albopictus* is one of the most invasive and widespread mosquito species in the world. Technological advances in mass production, overseas trade, and global travel have accelerated its movement within and across continents. One of the factors contributing to the spread of *Ae. albopictus* is its close association with human activities and dwellings, which has facilitated the movement of eggs around the world and resulted in the invasion of new lands with suitable climates. In California, it has been speculated that the hot, dry summer period typical throughout most of the state provides a hostile environment for the rapid population growth and establishment of this species [15], [16]. This assumption was initially supported by apparent inability of *Ae. albopictus* to permanently establish despite numerous opportunities, particularly during the extensive introductions from China discovered during the summer of 2001 [12], [35]. It was unexpected therefore when a relatively widespread inland population of *Ae. albopictus* was discovered in Los Angeles County in early September of 2011 in an area comprised primarily of single-family suburban homes [17]. With no potential links to national or international trade identified, the origin of this newly-discovered population was uncertain. The subsequent difficulty in detecting and controlling these mosquitoes within the infestation area fueled the need to identify the origin of this population to better understand its ecology and estimate how long it had been present in the area. This information would be helpful in determining the scope of surveillance and control measures needed for curtailing further spread and preventing future introductions, ultimately minimizing the potential public health impact.

The CO1 gene is a valuable diagnostic tool to study genetic diversity and spread of *Ae. albopictus* worldwide. The mitochondrial genome of *Aedes* mosquitoes is maternally inherited and very rarely undergoes recombination [36], thus reflecting more-or-less linear or clonal evolution compared to nuclear genes. In addition, the coding genes display a relatively rapid rate of evolution [36], [37] and have been shown to be useful in resolving inter-population relationships [38]. The CO1 gene has previously been used to establish intraspecific relationships of Mediterranean fruit flies [39] and *Anopheles* and *Aedes* mosquitoes [40], [41]. In this study, we detected a high level of polymorphism (66 haplotypes) among the CO1 sequences of the *Ae. albopictus* samples, which was much higher than that observed in other *Aedes* populations (≤4 haplotypes) previously reported in Cameroon [42]. A lower level of polymorphism in the Cameroon populations may be attributed to the recent invasion of *Ae. albopictus* into the country or the inclusion of samples from a relatively narrow geographical range [42]. By comparison, the greater number of haplotypes detected in our samples might partially result from the longer fragment of CO1 gene that was amplified and sequenced (>90% of the entire CO1 gene in length, i.e., 1433 of 1537 bp) and the wider geographic regions from which specimens were collected. Our sampling and analyses enabled us to determine the phylogeographic relationships of populations from various regions of Asia, Europe, and the U.S., and to infer the probable origin of the *Ae. albopictus* mosquitoes recently discovered in Los Angeles County.

The article "Genetic Analysis of Invasive Aedes albopictus Populations in Los Angeles County, California and Its Potential Public Health Impact" was published in 2013. Journal: PLoS One.

The pattern of pairwise genetic differentiation estimated from the CO1 sequence data indicated a significant level of structure among the populations of *Ae. albopictus* included in this study. While most of the genetic variation was found within populations, these populations appear to have reached equilibrium and that population size remains stable through time (Table 2; Fig. 3). Of the Asian samples, the Jiangsu (JS) laboratory strain was found to be the least genetically diverse, likely due to a small number of founders and subsequent inbreeding over time. Specimens collected from the different parts of mainland China (including the JS laboratory strain), Taiwan, and Japan showed little genetic differentiation among populations, but each were slightly genetically differentiated from those collected in Singapore. This suggested frequent gene flow among populations in the temperate (subtropical) zones (GZ, TW, and XM) and possibly reduced gene flow within tropical populations (SG). A plausible explanation for this difference is that temperate populations of *Ae. albopictus* more likely undergo photoperiodic diapause compared to tropical populations, a factor that could increase their chances for human-aided dispersal [4], [43] and contribute to gene flow over greater areas.

Samples collected from Los Angeles County in 2001 and 2011 were in most part genetically similar to those from south China (GZ and XM) and Taiwan, suggesting a temperate Asian origin (clusters 2 and 6 in Fig. 2). However, some of the preserved specimens collected in 2001 were also found to share an almost identical gene pool with that of the Singapore population, implying a possible tropical origin for these specimens. Similar heterogeneous origins have also been reported in *Ae. albopictus* from other parts of the world. For instances, populations from Cameroon were related to tropical rather than to temperate or subtropical groups based on CO1 polymorphism analysis [42]. The *Ae. albopictus* populations found in Represa do Congo and São Luis in Brazil formed a lineage paraphyletic to tropical southeast Asian lineages, i.e. Cambodia, Vietnam, and Thailand [44], [45]. The analysis of allozyme data revealed a close genetic association between the *Ae. albopictus* populations in the U.S. and Japan, implying a possible temperate Asian origin of the eastern U.S. populations [46]. These different conclusions with respect to the origin of *Ae. albopictus* illustrated the need for standardizing the method for mosquito sampling across its entire range as well as identifying more suitable genetic markers that can clearly and reliably establish the relationships among populations.

The article "Genetic Analysis of Invasive Aedes albopictus Populations in Los Angeles County, California and Its Potential Public Health Impact" was published in 2013. Journal: PLoS One.

The observed heterogeneity of gene pools among individual mosquitoes from Los Angeles County (both LA01 and LA11 specimens) implied multiple origins from different parts of Asia. Their genetic structures further suggested links to both temperate and tropical origins. Multiple introductions and origins of LA01 mosquitoes were likely since a tremendous number of *Dracaena* spp. plants arrived at the ports of Los Angeles and Long Beach in maritime containers for at least two years prior to the discovery in the summer of 2001 [35]. It was apparent that *Ae. albopictus* was using this cargo as an invasion pathway into California. Most *Dracaena* spp. originated from the temperate Guangdong Province in southern China (from where the genetically similar GZ specimens were collected), but plants were also grown and exported from Taiwan, Thailand, Indonesia, Cambodia, and Vietnam [35] providing possible sources of tropical *Ae. albopictus.* Multiple introductions have been critically important for invasive species such as *Ae. albopictus* to become established and in forming their population genetic structure [47]. In addition, multiple introductions may increase the genetic variation within a population over time, and in turn facilitate expansion and adaptation to novel environments. Founding populations of invasive species are commonly expected to experience severe genetic bottlenecks with reduced variation. However, this seems not to be the case for the two LA populations. Results of Tajima’s *D* and Fu’s *Fs* tests (Table 2) and the atypical shape of mismatched distribution (Fig. 3) indicated no sign of population bottleneck/expansion but in demographic equilibrium. Thus, these populations could have existed for sometime rather than recently invaded as a new founding population. It is very likely that the population currently present in Los Angeles County was founded during the 2001 introductions from southern China, and that the reduced proportion of Singapore gene pool in the LA11 collection implies the elimination of early-introduced tropical genotypes.

The article "Genetic Analysis of Invasive Aedes albopictus Populations in Los Angeles County, California and Its Potential Public Health Impact" was published in 2013. Journal: PLoS One.

The premise that LA11 may represent a carryover population is supported by empirical evidence and surveillance data collected in Los Angeles County following the initial detection of *Ae. albopictus* in 2001. The aggressive eradication campaign centered on infested wholesale nurseries was regarded a success at most locations; however, *Ae. albopictus* apparently survived the winter to reemerge in 2002 at two nursery locations and up to 500 m away in surrounding residential neighborhoods [13], [14]. Additional specimens were collected sporadically around one of these nurseries through July of 2004 suggesting persistence of this population in the environment (SK, unpublished data), but the lack of any further visual or trap-based evidence of mosquitoes was interpreted as confirmation that *Ae. albopictus* had been eradicated throughout the region. Two of the 15 wholesale nurseries discovered in 2001 were located in the City of El Monte [13], within the heart of the current infestation area of approximately 46 km^2^ [48]. It is possible that a small number of founder mosquitoes escaped detection due to the difficulty in sampling *Ae. albopictus* with available surveillance equipment. The region’s large population of immigrants who are native to countries where *Ae. albopictus* or other day-biting species are common and the patchy distribution of *Ae. albopictus* in neighborhoods lends credence to how this established population may have escaped detection for potentially over a decade [17], [48].

This study represents the first genetic analysis of *Ae. albopictus* invading California. The genetic data presented herein combination with earlier shipping records and local surveillance strongly support the notion that the population in the cities of El Monte and South El Monte was founded by individuals imported during the late 1990 s or early 2000 s from Asia. The size of the infested area suggests a relatively slow rate of spread that could be a result of the short dispersal range typical of this species [49], but might also provide direct evidence that while the southern California environment can support this species, it is less than ideal [15], [16]. Microhabitats present in heavily-irrigated residential properties and water-filled containers may provide the only suitable habitat for both adults and larvae and may explain their uneven distribution and variable abundance. Persistent control efforts with an emphasis on source reduction conceivably could prevent further spread and possibly results in either containment or eradication of *Ae. albopictus*. The inconsistent presence of adults observed throughout the infested neighborhoods creates a weak foundation for transmission of dengue or chikungunya viruses. Nonetheless, an established population of *Ae. albopictus* leaves open the potential for endemic transmission of these viruses in the area. The re-discovery of *Ae. albopictus* in Los Angeles County in 2011 provides convincing evidence that this species can become established in California and could become a severe nuisance and competent vector of disease. Local mosquito and vector control agencies should strongly consider including proactive surveillance and control programs for *Ae. albopictus* to maximize the potential for early detection and eradication.

The article "Genetic Analysis of Invasive Aedes albopictus Populations in Los Angeles County, California and Its Potential Public Health Impact" was published in 2013. Journal: PLoS One.

## Supporting Information

Table S1 **Sixty-six COI gene haplotypes identified in the 12** ***Aedes albopictus*** **populations examined.** Identity with the reference sequence (Genbank accession no. JQ004525) is denoted by a dot and substitution by a different base letter. GZ: Guangzhou; XM: Xiamen; JS: Jiangsu; TW: Taiwan; JP: Japan; SG: Singapore; IT: Italy; LA01: Los Angeles 2001; LA11: Los Angeles 2011; NJ: New Jersey; TX: Texas; and HW: Hawai’i.
(XLSX)
